RETRACTED

# Quantitative Relationship between the Degree of Lumbar Disc Degeneration and Intervertebral Disc Height in Patients with Low Back Pain

**DOI:** 10.1155/2022/5960317

**Published:** 2022-07-19

**Authors:** Jun Zheng, CaiLiang Shen

**Affiliations:** Department of Spine Surgery, The First Affiliated Hospital of Anhui Medical University, HeFei 230022, Anhui, China

## Abstract

The aim of this study is to study the relationship between the degree of lumbar disc degeneration and the height of the disc in patients with pain in the lower back and determine whether there is a dose-response relationship between the two. Eighty-five patients were examined by magnetic resonance imaging (MRI). The grade of lumbar degeneration was determined by the Pfirrmann grading system, and the intervertebral height and VAS pain scores were measured. The height difference of intervertebral discs with different degeneration levels was measured by the F test. This difference was correlated and further quantified by regression analysis. Finally, the differences intervertebral disc heights with a VAS score of 0–6 and 7–10 were observed by an independent sample *t*-test. The higher degree of disc degeneration in each lumbosacral segment, the lower the intervertebral disc height (*p* ≤ 0.011). When discs with grade 1 and grade 5 degeneration were excluded, the results remained the same (*p* ≤ 0.034). To quantify correlations, at each lumbar level, the disc height was reduced for each level of lumbosacral disc degeneration, and the height of disc was reduced after adjusting according to age, sex, and BMI (*β* range: −1.25 mm to −1.76 mm, 95% CI: −0.83 to −2.29, all *p* ≤ 0.002). Subjects with a VAS score of 7–10 had a lower intervertebral disc height than those with a VAS score of 0–6, especially with respect to total height levels at L4/5, L5/S1, and L1-S1 (*p* ≤ 0.04). This study showed a relationship between increased degree of intervertebral disc degeneration and decreased the disc height in patients with pain in the low back. Although the assessment of lumbar and lumbosacral level disc degeneration involves many qualitative measurements, these statistical data confirm the effectiveness of lumbosacral disc height as a continuous data measure and quantification in clinical trials and epidemiological studies.

## 1. Introduction

Epidemiological statistics have shown that [1] pain in the lower back is one of the biggest population health problems in the world, especially the elderly. With increasing economic and social development, the rate of pain in the low back in European and American populations has shown a yearly increase, which has exceeded that of spinal cord injury. The pain has the highest rate of disability. Teichtahl's study has confirmed a relationship between increased lumbosacral disc degeneration severity and decreased lumbosacral disc height in Australia [2]. China has also witnessed a yearly spike in the incidence of the pain, given the changes to working environment due to, economic development. Low back pain will inevitably cause heavy loss to the social economy of the country, especially considering the growing aging population. The pain after disc degeneration is more common in outpatients [3]. Lumbosacral disc degeneration means that long-term chronic low back pain is more likely and is twice as likely as it is without degeneration [4, 5], which will become an important direction of epidemiological research and the focus of our research.

RETRACTED

At present, in the literature, we have several understandings of intervertebral disc degeneration. Histological research mainly focuses on cartilage proliferation, degeneration, apoptosis, tear formation, and release of inflammatory factors [6]. The general macroscopic grading system includes changes in the morphology of the nucleus pulposus, fibrous rings, end plates, and vertebral bodies [7]. Clinically, intervertebral disc degeneration is classified by imaging of different degrees of intervertebral space stenosis, vertebral body deformation, hyperplasia of vertebral margins, and sclerosis of upper and lower endplates [8, 9]. The existing grading system of intervertebral disc degeneration showed that Pfirrmann's classification (2001) [9] is a widely used and recognized grading system for evaluating degree of intervertebral disc degeneration [10]. The Pfirrmann system is based on conventional magnetic resonance midsagittal T2-weighted image assessment using many qualitative features of MRI, including the nucleus pulp, the boundaries of nucleus pulposus and fibrous rings, signal intensity, and lumbar intervertebral height, and it is a 5 points grading system [10] (Figure 1). However, there is no mention of techniques for dynamically measuring disc degeneration, so it is hard to effectively detect dynamic changes in disc degeneration. Given that MRI would readily and quantitatively assess intervertebral disc height, our study would examine the relationship between the degree of lumbar intervertebral disc degeneration and the disc height in patients with lower back pain using the Pfirrmann grading system.

## 2. Materials and Methods

### 2.1. General Data

Patients with pain in the lower back and lumbosacral MRI examination were selected from the spinal surgery clinic of our hospital between April 2021 and June 2021. The exclusion criteria were as follows: (1) patients aged <25 years and >60 years; (2) patients with history of malignant tumor and obvious systemic diseases such as cerebrovascular accident, dyskinesia, or connective tissue disease; (3) those with a history of lumbar surgery; (4) those with wedge-shaped changes to the lumbar vertebrae, Modic changes, Schmorl's nodules in the intervertebral discs, and vertebral endplate abnormality; (5) those with pathological spinal injuries, such as bone tumor, spinal tuberculosis, and spinal infection; and (6) those who could not successfully complete an MRI scan owing to either claustrophobia or poor compliance. All patients provided written informed consent.

RETRACTED

### 2.2. Experimental Equipment

MRI was performed with a 3.0 T scanner (Prisma). All imaged were obtained with the patients in the supine position without changing position. The scanning details are as follows:

Sagittal images of T12 to T1 of the sacrum (repetition time: 490 ms, echo time: 8.8 ms, slice thickness: 4 mm); T2 sagittal images (repetition time: 2000 ms, echo time: 82 ms, slice thickness: 4 mm); T2 transverse axial (repetition time: 2500 ms, echo time: 89 ms, slice thickness: 5.5 mm).

### 2.3. Methods of Measurement

#### 2.3.1. Evaluation of Intervertebral Disc Degeneration

Pfirrmann's grading system [10] would be used to evaluate lumbosacral and lumbar intervertebral disc degeneration on T2-weighted sagittal images, as shown in Figure 1, and was measured by an experienced radiologist with MRI experience. Regardless of the characteristics of the subjects, the two groups of images were reevaluated after a one week interval. The reliability of intervertebral disc degeneration measurement was high at each lumbar vertebral level, and the intraclass correlation coefficient (ICCs) was between 0.89 and 0.96. The measurement of intervertebral disc degeneration showed high reliability at each vertebral level.

#### 2.3.2. Intervertebral Disc Height Measurement

T1-weighted middle sagittal MRI was used to measure the lumbosacral disc height. To ensure the accuracy of lumbosacral intervertebral disc height, the corresponding sagittal MR image was determined by adjusting the transverse axial scanning plane, and the image was enlarged 4 four times. From the middle of the upper edge to the middle of the lower margin of the intervertebral disc, there are two endplates. Intervertebral disc height was measured by an experienced MRI radiologist and remeasured at an interval of one week, regardless of the demographic characteristics. The results of intervertebral disc height measurement of each level were reliable, and the range of intraclass correlation coefficient (ICC) was 0.92–0.97.

#### 2.3.3. Anthropometric Data

The height measured with a rangefinder was accurate to 0.1 cm. We used a pair of electronic scales to measure weight up to 0.1 kg. the body mass index (BMI) (kg/m^2^) of each patient was calculated.

RETRACTED

#### 2.3.4. Visual Analog Scale (VAS) Measurement

The VAS is the most commonly used tool to measure pain intensity [11]. VAS in this study has high feasibility, low burden on researchers and subjects, is simple and intuitive, and easy scoring.

Zero points: painless; <3 points: slight pain, could endure; 4–6 points: pain could affect sleep, but could still endure; 7–10 points: gradually intensifying, unbearable pain that could affect appetite and sleep.

### 2.4. Statistical Methods

All analyses were performed by the SPSS statistical software (standard version 20.0 SPSS, Chicago, IL, USA). An F test would be used to determine whether the null hypothesis that the average disc height is uniform could be rejected. To rule out the overall effect of Pfirrmann grade 1 and grade 5 degeneration, subgroup analysis of grades 2–4 disc degeneration was reperformed. Linear regression analysis was used to determine the dose-response relationship between them and was adjusted according to age, sex, and BMI. Using a two-sample independent *t*-test, we compared patients with VAS scores >6 points (i.e., unbearable strong pain) and ≤6 points (i.e., the average height of the intervertebral disc can be tolerated by general pain). A *p* value of <0.05 was considered statistically significant.

## 3. Results

Demographic characteristics of 85 participants are shown in Table 1. There were 32 men and 53 women (mean age, 49.7 ± 7.8 years). Eleven men and 24 women were aged between 40 and 50 years, and 18 men and 26 women were aged between 50 and 60 years. The average BMI of participants was 28.5 ± 7.3 kg/m^2^. The number of degenerations in each lumbosacral segment corresponding to the degree of lumbosacral disc degeneration is also shown in Table 1. The overall performance at the L4/5 and L5/S1 level was more obvious with more severe grades at lumbar 45, lumbar 5 sacral 1 intervertebral disc segment. The average height (in mm) of the intervertebral discs of each lumbosacral segment was L1/2: 9.7 ± 1.1, L2/3: 10.8 ± 1.4, L3/4: 11.6 ± 1.6, L4/5: 11.3 ± 1.8, and L5/S1: 10.2 ± 2.2. We recorded 23 cases with VAS score >6 points and 62 cases with VAS score ≤6 points.

The box plot is more intuitive to show the relationship between the average height of the disc (*Y*-axis) and Pfirrmann grading (*X*-axis) of lumbar disc degeneration, as shown in Figure 2, which showed that the L1/2, L2/3, L4/5, and L5/S1 horizontal lumbar and lumbosacral disc height had a significant decline with the rise of disc degeneration level. As there were no discs with grade 1 and grade 5 degeneration at the L3/4 level, this change was not obvious.

RETRACTED

To distinguish this height change, the F test could be used to compare the different levels of intervertebral discs in each lumbosacral segment, as shown in Table 2. After regulating for age, sex, and BMI, the *p* values were ≤0.011, in order to ensure that sexual differences were not caused by grade 1 and 5 lumbosacral disc degeneration. In particular, there was an obvious loss of disc height seen in grade 5 degeneration. Subgroup analysis was performed again, and the results had not unchanged (grades 2–4 disc degeneration, *p* ≤ 0.034).

In order to quantify the relationship between them, statistical multiple linear regression analysis was used, as shown in Table 3. After adjusting for demographic characteristics, there would be a significant decrease in the height of disc in each lumbosacral segment (*p* ≤ 0.002):

L1/2: *β*,−1.25 mm (95% CI: −1.67 to −0.83); L2/3: *β*, −1.43 mm (95% CI: −1.82 to −1.04); L3/4: *β*, −1.66 mm (95% CI: −2.24 to −1.10); L4/5: *β*, −1.76 mm (95% CI: −2.29 to −1.23); and L5/S1: *β*, −1.61 mm (95% CI: −2.10 to −1.12).

The independent sample *t*-test compared the VAS scores of ≥6 points and ≤6 points for different lumbosacral disc heights, as shown in Table 4. At each lumbosacral disc level, the height of the intervertebral disc with a VAS score of 7–10 was lower than the height of the disc with a VAS score of 0–6, which was at the L4/5 (11.7 mm vs. 10.1 mm, *p*=0.01) and L5/S1 (10.5 mm vs. 9.5 mm, *p*=0.04) levels; the cumulative intervertebral disc height (54.9 mm vs. 49.7 mm, *p*=0.03) was also statistically significant.

## 4. Discussion

This study confirmed a significant negative dose-response relationship between the degree of L1-S1 disc degeneration and the height of lumbosacral disc in patients with pain in the low back. In particular, for each additional stage of lumbosacral disc degeneration, the narrowing range of the disc was 1.25–1.76 mm. Although there are several qualitative measures' assessment of disc degeneration, these statistical data confirm the effectiveness of disc height as a continuous data measure and quantification in clinical trials and epidemiological studies.

In this study, the Pfirrmann grading system was used to classify intervertebral disc degeneration. This grading system is an effective method for evaluating by MRI [10, 12]. In the Pfirrmann system, the lumbosacral disc height is divided into 5 grades. None of the measurements directly quantify the lumbosacral disc height; therefore, the definition of normal disc height within and among individuals is somewhat vague. However, in our study, the measurement of the height in patients with pain in the low back showed a significant decrease in lumbosacral disc height with each grade of degeneration. The level of disc in the lumbosacral segment ranged from 1.25 mm to 1.76 mm, regardless of age, sex, or BMI.

RETRACTED

In the Pfirrmann grading system, the only grade that contains a significant reduction in the lumbosacral disc height is grade 5. For example, at the L4/5 level, the average height was 10.12 mm for grade 4 degeneration and 5.56 mm for grade 5 degeneration. Similarly, at the L5/S1 level, the disc height in grade 4 regressed to 9.26 mm and that in grade 5 regressed to 5.61 mm. In addition, at the same segment of the lumbar disc, such as the L5/S1 level, the respective mean disc heights for grades 2, 3, and 4 disc degeneration were 11.79 mm, 10.66 mm, and 9.26 mm. For specialist practitioners who distinguish between the degree of lumbosacral disc degeneration, this small reduction in the disc height was unlikely to be visually identifiable. There was clear stenosis at each lumbosacral intervertebral disc level (all *p* ≤ 0.034). Urquhart et al. showed that the reduction of the lumbar disc height is associated with increased risks of pain in lower back [13]. This was confirmed in our study based on results that showed that the intervertebral disc height of subjects with VAS score of 0–6 was lower than that of subjects with VAS score of 7–10, especially in the total height levels of L4/5, L5/S1, and L1-S1. At the same time, in a case-control study, older patients with more degree degenerative lumbar disease had twice the risk of chronic pain than nondegenerative disc [4], and this finding was validated elsewhere [2, 5]. In summary, these results show that although assessment of generalized disc degeneration is based on qualitative methods, disc height—as a continuous measurement—can better identify disc degeneration, especially when there is no significant decrease in height; this can provide a potentially more sensitive quantitative assessment method for lumbar disc degeneration.

Furthermore, we quantitatively defined the height changes of intervertebral discs showing different degrees of degeneration using the Pfirrmann grading system. The further improved the evaluation of lumbosacral and lumbar disc degeneration by the Pfirrmann grading system, e.g., the Pfirrmann grading system defines grade 3 intervertebral disc height as slightly decreased and grade 4 height as moderately decreased. However, our data showed a moderate decrease in the height of level 3 and level 4 discs, and this difference was statistically significant. In addition, previous studies have pointed out that it may be difficult to classify elderly patients' spines using the Pfirrmann grading system (mean age: 73 years; age range: 67–83 years); accordingly, this grading system needs suitable modifications [14]. As the mean age of our patient sample was 49.7 ± 7.8 years, no modifications were necessary to the scoring and grading system. Finally, we noticed a significant change in disc heights of grades 1 and 5 degeneration, and a small sample cost may have biased the statistical results of our study. However, when subgroup analysis was performed after excluding the discs with grades 1 and grade 5 degeneration, the result remains the same. Equally important are the different statistical methods used in our study. We used *F* test to determine whether lumbar disc heights were consistent across different degrees of lumbosacral disc degeneration. However, this method cannot identify the direction of these differences. But these differences were quantified in linear regression analysis and illustrated graphically, as shown in Table 3 and Figure 2.

RETRACTED

Our study has some limitations. As this study included subjects with pain in the low back, which may led to an inadvertent bias in subjects with more severe lumbar and lumbosacral disc degeneration, essentially limiting generalizability of the findings to patients without low back pain. Therefore, further research is needed to address these issues.

## 5. Conclusion

Data from this study show a dose-response relationship between the degree of lumbar and lumbosacral disc degeneration and the height of disc. Although there are several qualitative measures' assessment of disc degeneration, these statistical data confirm the effectiveness of disc height as a continuous data measure and quantification in clinical trials and epidemiological studies.

## Figures and Tables

**Figure 1:** Pfirrmann grading of lumbar disc degeneration (2001) [10].

**Figure 2:** Intervertebral disc height and Pfirrmann grading box diagram (L1/2, L2/3, L4/5, and L5/S1 intervertebral disc).

**Table 1:** Basic demographic data of the subjects. These results were expressed as mean ± standard deviation unless otherwise stated.

Characteristics	Value				
*Age (years)*	49.7 ± 7.8				
*Sex, n (%) female*	53 (62.4)				
*Body mass index (kg/m * ^*2*^ * )*	28.5 ± 7.3				

*Disc degeneration grade, n* (%)	1	2	3	4	5

L1/2	1 (1.2)	59 (69.4)	20 (23.5)	5 (5.9)	0 (0)
L2/3	0 (0)	47 (55.3)	29 (34.1)	8 (9.4)	1 (1.2)
L3/4	0 (0)	32 (37.6)	43 (50.6)	10 (11.8)	0 (0)
L4/5	0 (0)	14 (16.5)	35 (41.2)	35 (41.2)	1 (1.2)
L5/S1	1 (1.2)	25 (29.4)	28 (32.9)	24 (28.2)	7 (8.2)

*Lumbosacral and lumbar disc height* (mm)					
L1/2	9.7 ± 1.1				
L2/3	10.8 ± 1.4				
L3/4	11.6 ± 1.6				
L4/5	11.3 ± 1.8				
L5/S1	10.2 ± 2.2				

*VAS score, n (%)*					
≤3	13(15.3)				
4–6	49(57.6)				
7–10	23(27.1)				

RETRACTED

**Table 2:** Intervertebral disc heights with different degeneration grades at each segment level (mean ± standard error).

	Intervertebral height of lumbosacral disc degeneration at different levels (in mm)						
	1	2	3	4	5	*P* ^a^	*P* ^b^
L1/2	12.51 ± 0.03	10.06 ± 0.4	8.74 ± 0.4	7.84 ± 0.4	—	0.009	0.034
L2/3	—	11.65 ± 0.5	9.98 ± 0.3	8.78 ± 0.4	6.16 ± 0.02	<0.001	0.001
L3/4	—	12.99 ± 0.7	10.98 ± 0.5	9.92 ± 0.5	—	0.011	0.011
L4/5	—	13.39 ± 1.0	11.74 ± 0.5	10.12 ± 0.6	5.56 ± 0.02	<0.001	<0.001
L5/S1	14.19 ± 0.04	11.79 ± 0.5	10.66 ± 0.6	9.26 ± 0.9	5.61 ± 0.8	<0.001	0.004

*P* value is *F* test two-two comparison maximum *P*^a^: Comparison of grades 1–5 disc heights; *P*^b^: Comparison of grades 2–4 discs.

**Table 3:** Relationships between the degree of lumbosacral disc degeneration (grade 2–4) and the intervertebral height (mm) of corresponding segments.

	*β*1 (95% CI)	*P*	*β*2 (95% CI)	*P*
L1/2	−1.26(−1.56, −0.96)	<0.001	−1.25(−1.67, −0.83)	<0.001
L2/3	−1.57(−1.84, −1.30)	<0.001	−1.43(−1.82, −1.04)	<0.001
L3/4	−1.68(−2.07, −1.29)	<0.001	−1.66(−2.24, −1.10)	0.002
L4/5	−1.74(−2.12, −1.36)	<0.001	−1.76(−2.29, −1.23)	0.001
L5/S1	−1.69(−2.02, −1.37)	<0.001	−1.61(−2.10, −1.12)	<0.001

*β*1: simple linear regression coefficient; *β*2: multiple linear regression coefficients after adjusting for age, sex, and BMI.

**Table 4:** Comparison of the VAS score 0–6 and VAS score 7–10 of intervertebral disc height.

	VAS score 0–6 *n* = 62 (72.9%)	VAS score 7–10 *n* = 23 (27.1%)	*P*
L1/2	9.8	9.2	0.19
L2/3	11	10.1	0.09
L3/4	11.9	10.8	0.07
L4/5	11.7	10.1	0.01
L5/S1	10.5	9.5	0.04
Cumulative L1-S1 disc height	54.9	49.7	0.03

## Data Availability

The simulation experiment data used to support the findings of this study are available from the corresponding author upon request.
